# Human Gait Analysis and Prediction Using the Levenberg-Marquardt Method

**DOI:** 10.1155/2021/5541255

**Published:** 2021-02-18

**Authors:** Abdullah Alharbi, Kamran Equbal, Sultan Ahmad, Haseeb Ur Rahman, Hashem Alyami

**Affiliations:** ^1^Department of Information Technology, College of Computers and Information Technology, Taif University, P.O. Box 11099, Taif 21944, Saudi Arabia; ^2^Biomedical Engineering, Vellore Institute of Technology, Vellore, Tamil Nadu 632014, India; ^3^Department of Computer Science, College of Computer Engineering and Sciences, Prince Sattam Bin Abdulaziz University, Al-Kharj 11942, Saudi Arabia; ^4^Department of Computer Science & Information Technology, University of Malakand, Chakdara Dir Lower, Pakistan; ^5^Department of Computer Science, College of Computers and Information Technology, Taif University, Taif 21944, Saudi Arabia

## Abstract

A high-accuracy gait data prediction model can be used to design prosthesis and orthosis for people having amputations or ailments of the lower limb. The objective of this study is to observe the gait data of different subjects and design a neural network to predict future gait angles for fixed speeds. The data were recorded via a Biometrics goniometer, while the subjects were walking on a treadmill for 20 seconds each at 2.4 kmph, 3.6 kmph, and 5.4 kmph. The data were then imported into Matlab, filtered to remove movement artifacts, and then used to design a neural network with 60% data for training, 20% for validation, and remaining 20% for testing using the LevenbergMarquardt method. The mean-squared error for all the cases was in the order of 10^−3^ or lower confirming that our method is correct. For further comparison, we randomly tested the neural network function with untrained data and compared the expected output with actual output of the neural network function using Pearson's correlation coefficient and correlation plots. We conclude that our framework can be successfully used to design prosthesis and orthosis for lower limb. It can also be used to validate gait data and compare it to expected data in rehabilitation engineering.

## 1. Introduction

In the entire world, there is an ever-increasing count of amputees. Spoden et al. established that in Germany alone, the number of lower leg amputation cases was 52,096 in 2005 and 55,595 in 2015, confirming that a significant population suffers from lower leg amputations and it is on the increase [1]. A study by Manickum et al. suggests that 53.1% of lower leg amputations are caused by Diabetes Mellitus alone [2]. In India, Pooja et al. performed a study of 155 amputees and observed trauma to be the primary cause of amputation (70%) followed by vascular diseases. They also reported 94.8% of all amputations were of the lower limb [3]. The people having amputations have a very peculiar and different gait cycle as compared to an average human, which makes them unconfident about themselves, driving them towards depression and anxiety [4] because of pain and pity. The primary target of any commercial prosthesis or orthoses is to reduce the gap between the gait data of its user and that of a healthy adult of the same physiology. Human gait refers to the walking pattern of Homo sapiens. It is similar for all healthy human adults and comprises different continuous phases in order, such as Heel Strike, Loading Response, Mid Stance, Terminal Response, and Swing Phase (Preswing and Swing). While designing and constructing a prosthesis (lower or upper limb), the primary aim is always to make it as similar as possible to that of a healthy person, which is why the data recorded from a healthy human still act as a reference for such purposes. Nowadays, there is always the demand for a more and more intelligent and active prosthesis (working on an energy source) rather than a passive prosthesis (without an energy source). In general, the training time required by the patient to adjust to an active prosthesis is higher than that needed for a passive prosthesis. Yet, they are of higher demand because of their better performance aspect. The only other major drawback with active or adaptive prostheses/orthoses is their design complications. To simplify this, Chan et al. came up with an EMG based gait phase prediction model for prosthesis control [5]. As an extension of their work, Lee and Lee proposed the technique for predicting the posture angles of the patient's orthosis for a single lower limb [6]. Moissenet et al. tried the regression model approach to determine deviations for physiological and pathological subjects; however, we kept our study limited to perfectly healthy subjects [7]. Recently, Kim et al. used Doppler radar data for human gait analysis [8]. In this paper, we propose a neural network-based prediction control scheme for intelligent orthoses and prostheses, where the gait data for the next 20 seconds are predicted for given constant speed. In the case of Lee and Lee, the error was approx. 0.5°, but in our neural network model, the error (MSE) is in the order of 10^−4^. The oldest research work that could be traced in the field of gait pattern identification was done by Murray et al. in 1970 when they compared the gait data of women [9]. Muro et al. compared the accuracy of nonwearable and wearable sensors [10]. In a nutshell, it can be concluded that the gait data can be measured via wearable goniometric sensors as well as nonwearable image processing alternatives. The recent advancement in technology allows both these approaches to have a very good amount of accuracy. Yao et al. have already confirmed that gait data angles are similar for subjects, so long as they are walking, regardless of whether on a treadmill or over-ground [11]. Pardasani et al. presented an algorithm for using the Kinnect-based mocap procedure for comparative analysis of gait data using a nonwearable sensor [12]. There have been several other recent published works on Kinnect and other nonwearable sensors [13, 14], but the scope of wearable sensors which can give much higher accuracy compared to nonwearable sensors is very limited. Internet of Things and its Sensors Devices are playing a great role in the new smart healthcare sector [15]. In this paper, first, we have presented basic information about human gait and its various stages and then discussed out data recording protocols and algorithm for designing neural network. The flow of the processes is as given in Figure 1.

## 2. Features of Human Gait

The human gait is a cycle of alternative forms of the lower limb, e.g., both the arms will always have the opposite form of each other while the subject is walking. This cycle is initiated when the foot of either leg hits the ground after a swing, called heel strike, and ends at the next heel strike of the same foot [16]. The various forms in between are loading response, midstance, terminal stance, preswing, and swing phase (preswing phase is mostly clubbed with the swing phase [17]). The loading response, midstance, and terminal stance can be collectively termed as support phase or stance phase. Gait comprises of alternative repetition of these two (swing and stance) phases, one after the other, tracing a continuous cycle. It is evident from Figure 2, and it has been demonstrated by Kour et al. [18] and Vaughan et al. [19] in their work that human gait continuously changes in angles of the hip joint, knee joint as well as ankle joint. These changes are brought about by the energy gradient in the human skeletal muscles of the lower limb [20, 21].

## 3. Data Recording

Data were recorded for 5 different healthy subjects, able-bodied, without any known physiology or pathology at the time of recording. Sampling frequency was set at 100 Hz, i.e., 100 samples/second. The subjects were made to walk on a treadmill at following three constant velocities: 2.4 kmph (0.67 m/s), 3.6 kmph (1 m/s), and 5.4 kmph (1.5 m/s). Data were recorded at each of these speeds for 20 seconds each, keeping a buffer of 20 s at the start and between two consecutive recordings allowing sufficient transition time for the treadmill to gain the required velocity and the subject to acclimatize to the speed. The same steps were repeated for three instances per individual to ensure good quality of data is collected for analysis. So, a total of 45 different datasets were derived overall, which were then bifurcated into their respective speeds. Gait data were collected using the Biometrics goniometer. Data were recorded for each of the joints of both the lower limbs, i.e., right hip, left hip, right knee, and left knee. These subjects were aged 19–23 and weighed around 65–85 kgs, i.e., they were neither too obese nor too malnourished. A random subject during data recording can be seen in Figure 3. The location of the sensors is marked in black.

## 4. Methodology

As mentioned above, the data were recorded for five different healthy subjects, thrice for three different speeds, making it a total of 45 instances. Recorded data were first split based upon respective speeds because the device used to record the angle data using a Biometrics goniometer [22] exports the recorded data in a single file with each joint as a separate channel. A periodogram showed that they all had high-frequency noises in them, which was clear from the plot [23]. This noise can be attributed to the electronics involved and minute shifting of sensors while in motion. The actual data are only in the range of 0.5–5 Hz at maximum. So, appropriate low pass Butterworth filters were designed and applied to ensure the data can be made as much noise-free as possible. The most observable noises were the high-frequency noise observed from the spectrogram, as well as some aperiodic low-frequency noise, which was affecting the peaks of the signal. So, Butterworth low pass filters were used to filter out the high-frequency noise and preserve the low-frequency components, which too consisted of some noise as peak distortion was still observable in some cases. We have processed the different stages as the flow of the processes, available in Figure 1. So, to take care of that, a moving average filter was used with varying window sizes based upon the speed at which the subject is walking. But, for two different subjects, the window size applied was kept the same to ensure uniformity. Similarly, the low pass filters were designed separately for each speed, although it was kept the same for different individuals at the same speed. The several sets of figures (Figures 4–9) show before (b) and after filtration data (a) for 7 seconds for visualization purposes. Figures 4 and 5 for hip and knee, respectively, show the data at 2.4 kmph, Figures 6 and 7 at 3.6 kmph, and Figures 8 and 9 at 5.4 kmph.

Once it was done on the data recorded from all the subjects, it was observed that, although the signal of angle measurement at different speeds was slightly similar, at a constant speed, it was pretty identical not only in the three instances of the same subject but also in case two distinct subjects. So, we tried to train a neural net to design a function in Matlab, which will give the next angle if the previous 100 aspects recorded are given to it as an input (keeping in mind *f*_*s*_ = 100 Hz). This function can be used as a reference for designing prosthesis as well as validating gait in case of biomechanical rehabilitation. So, using a for loop for each data sequence recorded, two matrices were created, one to act as input for the neural net and the second one to serve as a target. These matrices were made for each speed separately so that separate networks can be trained to result in distinct functions for each speed. In the input matrix, every set of 101 consecutive cells was passed as one element from the data recorded and the 102^nd^ data were passed into the target matrix. This process was repeated for each individual at each speed. Afterward, the neural net was designed and trained. The algorithm used was the LevenbergMarquardt method using the Neural Network Toolbox of MatLab 2018a [24]. It was observed that after training the net only for the first subject, the functions were able to predict the data accurately for the remaining four subjects without even being trained by their data. For example, in the two plots shown in Figure 10, the one on top is the actual data recorded for the second individual and the one on the bottom is the neural net output although; it was trained only on the data of the first person. This particular data is of right hip, but a similar phenomenon has been observed in all the joints.

The uncanny similarity (as one of the plots almost superimposes the other) is further confirmed by correlation analysis calculated by Pearson's correlation coefficient, which proves that these two plots are exactly similar discussed later in the paper. The correlation coefficient, which is used to determine the similarity of two datasets scientifically, in this particular case, comes out to be 0.999, where affinity towards 1 suggests similarity and resemblance towards 0 suggests nonsimilarity of the data. In some cases, the coefficient can be negative, which suggests the two inputs being similar out of phase.

## 5. Neural Net Specifications

As mentioned earlier, using Matlab's Neural Net Fitting tool [24] and the abovementioned dataset and targets, separate neural nets were designed for each joint, and a Matlab code was exported using the same tool for function. The specific reason for using LM is that our data here are nonlinear, and the best approach to predict nonlinear data is to use the LM method. A total of 1600 samples were obtained for each case, out of which 1120 samples were used for training, 240 for testing, and 240 for validation in each case. Following individual functions were realized for each speed (2.4kmph, 3.6kmph, and 5.4 kmph separately):

(1) Right hip
  (1.1) Right hip slow, 2.4 km/h
  (1.2) Right hip medium, 3.6 km/h
  (1.3) Right hip fast, 5.4 km/h
(2) Left hip
  (2.1) Left hip slow, 2.4 km/h
  (2.2) Left hip medium, 3.6 km/h
  (2.3) Left hip fast, 5.4 km/h
(3) Right knee
  (3.1) Right knee slow, 2.4 km/h
  (3.2) Right knee medium, 3.6 km/h
  (3.3) Right knee fast, 5.4 km/h
(4) Left knee
  (4.1) Left knee slow, 2.4 km/h
  (4.2) Left knee medium, 3.6 km/h
  (4.3) Left knee fast, 5.4 km/h

It was then observed that the neural net showed unsupervised learning, and even if the net was trained for just one subject's data, it was able to predict the data for the remaining subjects accurately. However, they were never trained for that subject. Furthermore, the accuracy was so high that the correlation coefficient was always in the range of 0.99. This can be accredited to the low mean-squared error while training the net. Roughly, every net had 1600 sets of inputs and targets. They were trained using LevenbergMarquardt Model as mentioned earlier, and the number of hidden layers was set between 10 and 25 determined by the hit and trial method wherever it gave the best output with maximum accuracy while not requiring a very long time to train the net, although still training each net took approx. 20–25 minutes. The intention was to establish an efficient tradeoff between accuracy and time required to train the model. Still, in most cases, the MSE was very low (Figure 11(a)), so the figure was settled at ten although it may vary depending upon the initial conditions and the output accuracy. The exact time could vary based upon the initial conditions which are taken randomly in the case of the LM Model. The very low mean-squared error resulted in a very high correlation coefficient, which proves the high accuracy of the net and the model. Figure 11(b) and 11(c) show the properties of the neural net designed.

## 6. Results and Validation

The neural net result was validated using the correlation coefficient and correlation plot to identify the similarity between the expected output and the corresponding neural net function output. These correlation plots have been plotted for both the dataset used for training as well as the dataset not used for training. Yet, the similarity is very high in both cases, confirming unsupervised learning of the neural net.  Table 1 shows the accuracy when the dataset used in training and the dataset used for validation are of same subject but from different trials.  Table 2 shows the accuracy when the dataset for training and validation belongs to two different subjects. Figures 12 and 13 show the correlation plot between the expected and the actual output of neural net function for right hip and right knee, respectively, at 3.6 kmph when the data belong to same subject but from different trials. Figures 14 and 15 show the same plots when the dataset belongs to two different subjects.

  Case-I: when training dataset and validating dataset are of same subject
  Case II: when training dataset and validating dataset are of different subjects

## 7. Conclusion

The study aims at proposing a new approach for prediction of gait data to be used for reference while designing prostheses and orthoses as well as validation of gait data during biomechanical rehabilitation. Experimentally, the least accuracy observed was 97.39% for a subject whose data are used to frame the model, whereas 96.54% for a subject whose data were not used to frame the model. Thus, we conclude our experiment to be a success. The prostheses and orthoses using this method are expected to have a very positive effect on the life of subjects and are likely to assist in the betterment of the quality of life of an amputee.

## Figures and Tables

**Figure 1:** Flow of the processes.

**Figure 2:** Various stages of human gait [18].

**Figure 3:** A random subject during data recording.

**Figure 4:** A Raw data of hips at 2.4 kmph (a) and filtered data of hips at 2.4 kmph (b).

**Figure 5:** Raw data of knees at 2.4 kmph (a) and filtered data of hips at 2.4 kmph (b).

**Figure 6:** Raw data of hips at 3.6 kmph (a) and filtered data of hips at 3.6 kmph (b).

**Figure 7:** Raw data of knees at 3.6 kmph (a) and filtered data of knees at 3.6 kmph (b).

**Figure 8:** Raw data of hips at 5.4 kmph (a) and filtered data of knees at 5.4 kmph (b).

**Figure 9:** Raw data of knees at 5.4 kmph (a) and filtered data of hips at 5.4 kmph (b).

**Figure 10:** Comparison between neural net output and expected output for the hip @3.6 kmph.

**Figure 11:** Neural net training specs for right hip @ 3.6 kmph.

**Figure 12:** Plot of correlation between neural net output and target for right hip at 3.6 km/h. The *Y*-axis is in the range of 10^5^ which confirms very high similarity in both the arrays passed.

**Figure 13:** The plot of correlation between neural net output and target for right knee at 3.6 km/h. The *Y*-axis is in the range of 10^5^, which confirms very high similarity in both the arrays passed.

**Figure 14:** Plot of correlation between neural net output and target for right hip at 3.6 km/h. The *Y*-axis is in the range of 105 which confirms very high similarity in both the arrays passed.

**Figure 15:** Plot of correlation between neural net output and target for right knee at 3.6 km/h. The *Y*-axis is in the range of 105, which confirms very high similarity in both the arrays passed.

**Table 1:** Percentage correlation values of output compared against the target for the dataset used for training.

Speed (kmph)	2.4	3.6	5.2
Correlation of right hip	99	100	100
Correlation of left hip	100	100	100
Correlation of right knee	99.33	97.39	98.03
Correlation of left knee	99.33	97.39	98.03

**Table 2:** Percentage correlation values of output compared against the target for dataset not used for training.

Speed (kmph)	2.4 (%)	3.6 (%)	5.2 (%)
Correlation of right hip	99.33	97.39	98.03
Correlation of left hip	100	100	100
Correlation of right knee	98.99	98.01	99.60
Correlation of left knee	98.86	96.54	98.87

## Data Availability

The data used to support the findings of this study are available from the corresponding author upon request.
